# Periapical Healing following Root Canal Treatment Using Different Endodontic Sealers: A Systematic Review

**DOI:** 10.1155/2022/3569281

**Published:** 2022-07-08

**Authors:** Akshay Khandelwal, Krishnamachari Janani, KavalipurapuVenkata Teja, Jerry Jose, Gopi Battineni, Francesco Riccitiello, Alessandra Valletta, Ajitha Palanivelu, Gianrico Spagnuolo

**Affiliations:** ^1^Conservative Dentistry and Endodontics, Gajanan Clinic, Kolkata, 700025 West Bengal, India; ^2^Department of Conservative Dentistry and Endodontics, SRM Dental College, Ramapuram, 600089 Chennai, India; ^3^Department of Conservative Dentistry and Endodontics, Mamata Institute of Dental Sciences, Bachupally, Hyderabad, 500090 Telangana State, India; ^4^Department of Conservative Dentistry and Endodontics, Saveetha Dental College & Hospitals, Saveetha Institute of Medical & Technical Sciences, Saveetha University, Chennai 600077, India; ^5^Clinical Research Centre School of Medicinal and Health Product Sciences, University of Camerino, Camerino 62032, Italy; ^6^Department of Neuroscience, Reproductive and Odontostomatological Sciences, University of Naples, Naples 80138, Italy

## Abstract

The healing of the periapical tissues is crucial to the success of root canal treatment. The review studies effectively examine various endodontic root canal sealants in terms of periapical healing. This systematic review was formulated following the PRISMA 2020 guidelines and registered in the international prospective register of systematic reviews (PROSPERO) number-CRD42021239192. To find relevant articles, PubMed Central and Medline databases (until February 2022) were searched. Studies that evaluated healing following the application of different endodontic sealers were analysed. A primary outcome measure was the resolution of periapical lesions following the endodontic treatment. In vivo studies comparing radiographic treatment outcomes and articles with a minimum of 6-month follow-up were included. A total of 9 clinical trial studies that met all the inclusion criteria were included in the analysis. The overall risk of bias was high in four studies out of nine studies. Periapical lesions showed significant healing after endodontic treatment regardless of sealer type, although bioceramic and bioactive sealers had shown better results.

## 1. Introduction

Periapical lesion results from an inflammatory response to microorganisms around the tooth root and the root canal [1]. It is an unpleasant consequence of a body's protective response to microorganisms from the infected root canal system, which causes chronic inflammation. Trauma, caries, or tooth wear are some of the common causes of periapical radiolucencies [1]. After the pulp tissue loses its blood supply as a result of trauma, microorganisms may colonise it, leading to periradicular pathosis. Before treatment, periapical lesions must be diagnosed, and endodontic status needs to be assessed. Endodontic treatment intends to lower the bacterial load as much as possible, with the lesion disappearing as a result [2]. Radiographically interpreted lesions are used to assess periapical inflammation. Evaluation of the periapical status and endodontic therapy by the periapical index (PAI) is reliable [3]. Successful endodontic treatment relies on proper instrumentation, comprehensive disinfection, and obturation.

The synergistic combination of the obturation material and the sealer creates a hermetic seal [4, 5]. An effective seal will prevent any future pathologies due to the prevention of bacterial proliferation. A root canal sealer should possess adequate biological, physical, and chemical properties [6, 7]. The effectiveness of the treatment is dependent upon the type, and composition of the sealant that makes one sealer superior to the other [6–9]. When in contact with the periradicular tissue, sealers release various substances, causing different reactions [7].

Studies have shown extensive giant cell response in the periapical area to calcium hydroxide-containing sealers [10]. This leads to a better reduction in microbial infection in a periapical area, promoting healing. In [11], the authors evaluated the healing histologically after root canal treatment using sealapex, calciobotic root canal sealer (CRCS), and apexit. They concluded that sealapex showed the maximum mineralized tissue deposition. The differences in the inflammatory responses elicited by calcium hydroxide-containing sealers might be the reason for the better outcomes obtained in previous animal studies. Animal experimentation had shown favourable results when the calcium hydroxide was placed in close contact with the living tissues [12]. Sealapex induces a pronounced differentiation of macrophages and giant cells. The release of calcium ions might be the reason for cell differentiation and macrophage activation. Case reports on the usage of sealapex sealers have demonstrated healing periapical lesions though there was an accidental extrusion beyond the apex [13]. Several reasons attribute to the healing of periapical lesions at different rates. Improper elimination of bacteria from root canal complex structures like an isthmus, open dentinal tubules, or lacunae of cellular cementum around the apical foramen can be one. Another reason can be an extrusion of infected dentin debris during mechanical instrumentation [14]. So, it is challenging to eliminate confounding factors when evaluating periapical healing. In routine clinical practice, clinicians employed a variety of sealers such as zinc oxide eugenol-based sealers, resin-based sealers, and calcium hydroxide-based sealers [15]. With the advent of bioactive materials, the literature showed enhanced healing of periapical healing [16]. To address this, the present review analysed the periapical healing after root canal treatment using different root canal sealers.

## 2. Materials and Methods

### 2.1. Eligibility Criteria

A clinical trial and a randomized clinical trial comparing zinc oxide eugenol with other sealers in teeth with periapical lesions requiring root canal treatment were considered for inclusion. Studies that had a follow up of minimum of six months were recruited for this review. Full-text articles in the English language were included. A case report or case series, *in vitro* study, animal studies, or reviews containing open apices are excluded.

### 2.2. Information Source

A search strategy was developed to identify studies for this review in the PubMed, Scopus, and Cochrane database of systematic reviews and Google Scholar databases until the end of February 2022. Additionally, the reviewers checked reference lists and performed a manual search to eliminate the possibility of additional data. The search protocol has been registered in PROSPERO which is an international prospective register of systematic reviews (CRD42021239192).

### 2.3. Search Strategy

The document search was conducted using search terms such as “root canal treatment,” “endodontic treatment,” “bioceramic sealer,” “AH 26 sealer,” “zinc oxide eugenol sealer,” “AH plus sealer,” “resin sealer,” “calcium hydroxide-based sealer,” “bioceramic sealer,” and “periapical healing.”

### 2.4. Selection Process

Study population is patients with periapical lesions undergoing root canal treatment, intervention is zinc oxide eugenol (ZOE) based sealers, comparison is various endodontic sealers compared, and outcome is periapical healing evaluation. Epoxy resin-based sealers, silicone-based sealers, chloroform-based sealers, calcium hydroxide-containing sealers, mineral trioxide aggregate- (MTA-) based sealers, and bio ceramic-based sealers were included for assessment. Radiographic assessment was used to determine the degree of healing following root canal treatment with different endodontic sealers.

Based on this, the studies were reviewed by three investigators to screen the title and abstract (A.K, K.J., and K.V.T.). Following which full text articles were evaluated to determine thier eligibility and discussed with the fourth investigator (A.P.)

### 2.5. Data Collection Process

Further, two colleagues evaluated independently the included articles. For evaluating the final article selection, we used the Preferred Reporting Items for Systematic Reviews and Meta-Analyses (PRISMA) 2020 guidelines.

### 2.6. Data Items

Information such as study design, sample size, tooth type, study groups, types of sealer used, clinical protocol, outcome, evaluation methods, and follow up was recorded.

### 2.7. Risk of Bias

The Cochrane Risk of Bias Tool (RoB 2.0) was used to assess the risk of bias. Reports should include procedures for randomization, deviations from the intended interventions, lack of data on the outcome, measurement of the outcome, and the selection of the reported results.

## 3. Results

### 3.1. Search Outcomes

68 articles were identified in the electronic search, and 27 were excluded after reading the title abstract since they did not correspond with the outcomes of the study. Finally, 31 articles were fully considered for further analysis. We excluded 22 articles due to nonavailability of full text and noncompliance with the eligibility criteria; nine articles that met all eligibility requirements were included (Figure 1).

### 3.2. Study Characteristics

Study characteristics and experimental results are summarized in Tables 1 and 2.

#### 3.2.1. Sample Size

Although all included studies had mentioned the sample size of the population, there were no details regarding the method of sample size estimation and also the power of the study [17–25]. Except for one study [23], none of the cited articles reported on inflation of the sample size to compensate for the loss of follow up in the follow-up study. The sample size varied ranging between 45 and 571 participants in the included studies.

#### 3.2.2. Study Year

Four studies were published at least 20 years before [19–22]; two are not indexed [12, 13]. Possibly, only two studies have been published in recent years [23, 24].

#### 3.2.3. Statistical Analysis

All studies have reported on the statistical test employed in their study, whereas, in one study, there were no details of the statistical analysis employed [18].

#### 3.2.4. Types of Sealer

Based on the sealers' usage, three used AH 26 [18, 23, 25], two used AH plus [18, 23], and two used MTA [18, 25]. Alternately, two studies used calcium hydroxide CRCS [18, 22], two studied salicylate-based sealer [17, 22], three studies used bio ceramic sealer [13, 18, 19], and two studies used ProcoSol and Kloroperka [19, 20].

#### 3.2.5. Outcome

One study investigated other clinical symptoms such as a sinus tract, swelling, and mobility [18], and three studies evaluated the primary outcome of periapical healing [18, 23, 25]. Bardini et al. assessed the periapical healing after primary and secondary root canals [24].

#### 3.2.6. Follow-Up

In the evaluation of the follow-up duration, three studies had a follow-up period of six months [18, 23, 25], two had a follow-up period of 1 year [21, 24], one had a follow-up period of 3 years [14], and three had a follow-up period of 4 years [17, 20, 22]. Despite this, three of the included studies did not report the loss of follow up [17, 18, 25].

#### 3.2.7. Type of Teeth

The included studies in this review used single-rooted teeth in three studies [18, 23, 25], and another three used both anterior and posterior teeth [19, 20, 24]. The types of teeth included in the two studies were not mentioned [12, 17]. Until Huumonen et al., there had only been one study that evaluated single-rooted teeth and a single canal in a posterior tooth [21]. It is not clinically reliable to compare periapical healing when there is a lack of homogeneity in the selection of teeth included in the analysis. Different types of teeth have apical ramifications and apical deltas, which are different from one another. There is no homogeneity in the types of teeth used in all the studies as both anterior and posterior teeth were included. Although the apical ramification differs between anterior and posterior teeth [26], it can greatly influence the rate of healing with three-dimensional disinfection as it is one of the confounding factors.

#### 3.2.8. Single/Multivisit Treatment

Out of all the included studies, four did not mention the number and time of visits for obturation [17, 20, 22, 24]. In one study, root canal treatment was completed in one visit [18], while in other studies, it was completed in two visits. Except for two studies [18, 23], all studies assessed periapical healing with the periapical score index (PAI). Five other studies analysed radiographic examinations using digital radiographs and periapical index scores [17, 18, 20, 23, 24], while one used software for analysis [25]. Three studies used the relative to an identified distribution (RIDIT) score for analysis [18–20]. Nagar and Kumar [18] performed single visit endodontic treatment, whereas four other studies completed the treatment in two visits [19, 21, 23, 25]. Four studies did not mention the time of obturation [12, 15, 17, 19]. During the interappointment visit, the quality of the coronal seal influences the sterilization of the root canal. It was not mentioned in any of the included studies what type of interim restoration was used.

#### 3.2.9. Quality of Apical Seal

Four studies have performed lateral compaction [21–23, 25], and one study [24] performed warm vertical compaction whereas the remaining studies did not mention the method of obturation. It is equally critical to fill the root canal three-dimensionally as it is to disinfect it three-dimensionally. It is the opinion of the authors of the present systematic review. This is because a compromised apical seal may lead to an adverse outcome in teeth with a breached apical foramen. Apical obturation limits are a very influential factor that determines periapical healing prognosis. Unfortunately, none of the studies has reported the extent of obturation. Although it has been reported in a previous study [27] that, despite using biocompatible sealers such as MTA, however, when the sealer extended beyond the apex, it interfered with healing.

### 3.3. Risk Bias

The randomization process was not mentioned in three of the nine studies [17, 18, 22]. There were no deviations from the intervention in seven studies [19–25]. In one study, the outcome data were reported without mention of relative to an identified distribution (RIDIT) scores [17], and two studies reported no information regarding clinical signs and symptoms [17, 22]. Whereas one study reported some concerns in missing outcome data [18], four reported with measurement concerns in data outcome [17, 18, 21, 24], and three reported with low risk of bias in selective reporting [19, 20, 23]. Therefore, when assessing the overall risk of bias, it was found that four out of nine studies showed a high risk of bias [17, 18, 21, 24]. This review maintains a standard bias of low quality for the included studies (Figure 2).

## 4. Discussion

Healing of the periapical healing lesion depends on various factors starting from biomechanical preparation, disinfection of the root canal system, intracanal medicaments, type of root canal sealers, overzealous sealer extrusion, and apical extent of obturation. In the present review, the authors intend to evaluate the healing ability of different endodontic sealers following root canal treatment. The present systematic review discusses mainly the different types of sealers and the influential role of disinfection, biomechanical preparation, and impact due to extrusion of sealer.

### 4.1. Irrigation Protocol

In MTA based sealers, irrigation protocol is particularly significant, since EDTA interferes with hydration and affects microstructure [28]. MTA-based sealers have been used in two studies, and EDTA has been used as a chelating agent to remove the smear layer. However, no information was provided regarding the measures taken to overcome the sealing ability [18, 25]. Five studies out of nine did not mention the irrigation protocol [17, 19–22]. Studies have also shown that sealing ability is affected by the setting time of the sealers [29].

### 4.2. Biomechanical Preparation

The majority of the included studies did not report the size of the canal preparation, except for two [21]. According to one study, the apical preparation size was 35, but there was no information on the taper size [19]. Another source estimates canal preparation size at 30.07 [24]. The most critical factor in treating the periapical lesion is optimizing the shape of the canal biomechanically. This is to ensure a sufficient penetration of irrigants into the apical third of the root canal system [30]. A canal that is insufficiently shaped might lead to unsatisfactory healing of microbial load. Periapical healing might also be affected by this factor.

### 4.3. Foramen Violation and Instrumentation

An additional factor to consider is the violation of the apical foramen. In this manner, the root canal filling material adapts to root canal filling material challenges that might eventually compromise the apical seal, resulting in apical leakage. In addition, over instrumentation might result in infected debris being extruded beyond the apex. In two of the studies, hand instruments were used to shape the canals [19, 22], and the canals were prepared with reamers and H files by Eriksen et al. [19]. Three studies [23–25] used rotary instruments; four studies [17, 18, 20, 21] did not report the instruments or instrumentation techniques.

### 4.4. Sealer Extrusion

By establishing an accurate working length with hand instrumentation, debris extrusion is reduced when compared to rotary instrumentation. Biomechanical preparation is one of the major factors that contribute to periapical healing. Periapical healing is interfered with by debris extrusion and bacteria. Acute inflammation occurs in the periradicular tissues when microorganisms are extruded apically. As the number of bacteria increases (quantitative factor), so do the pathogenicity and virulence of the bacteria (qualitative factor). Therefore, it is imperative to emphasize that apically extruded bacteria are clinically significant.

Poor bacteria removal may be seen in root canal complex structures such as an isthmus, open dentinal tubules, or lacunae in the cellular cementum around the apical foramen. Infected dentin debris could also be extruded during mechanical instrumentation [28]. When evaluating periapical healing, it can be difficult to eliminate confounding factors. Additionally, all studies included in the present review assessed healing with a periapical and digital radiograph. Radiography of the periapical area cannot predict the outcome of endodontic treatment. Cone-beam computed tomography (CBCT) can be used for long-term longitudinal studies with strict evaluation criteria, as this review has indicated [31].

### 4.5. Comparative Studies

According to previous studies, AH plus can be used as a root canal sealer to improve periapical healing. There is evidence that when sealers are extruded beyond the apex, macrophages phagocytose them and do not affect periapical healing negatively [32]. Additionally, it is influenced by the physical, chemical, and solubility of the material. According to the literature review, resin-based sealers that are extruded beyond the apex require more time to resorb. It has been reported that radiographic visualization takes 10-16 years [33]. Calcium hydroxide plays an active role in teeth with apical periodontitis. As an intracanal medicament, it is effective against both anaerobic bacteria and bacterial lipopolysaccharides [34]. An earlier study compared calcium hydroxide sealers with other sealer types and analysed their ionization. Their study found that sealapex has significantly higher alkalinity and calcium release values when compared to CRCS, APEXIT, and sealer-26 sealers [35]. Two included studies in our systematic review [17, 22], which used CRCS and sealapex, did not corroborate the above results. Over four years, there were no significant differences between the groups.

In an open root apex, a calcium silicate MTA sealer was reported to block and prevent any apical fluid flow and to achieve a more stable and durable seal than traditional zinc oxide and calcium oxide containing sealers. This bioactive apical barrier is created due to the release of calcium ions and the formation of apatite deposits [36, 37], doi:10.5301/jabfm.5000162. Calcium silicate MTA cements when comes into contact with simulated body fluids like HBSS, it forms an apatite coating on the surface. This apatite layer may aid in improving biological activity at the periapical level of the bone by boosting barrier development and stimulating apical cell activation and differentiation [38]. doi:10.5301/jabfm.5000162. The percentage of sealer penetration around the canal perimeter has clinical significance because it represents the sealer's capacity to seal against microorganisms in the dentinal tubules, regardless of the sealer's depth of penetration [39]. doi:10.5301/jabfm.5000162

The Bioroot RCS sealant is considered a bioactive sealant. In comparison to bioceramic sealers, bioactive sealers have been reported to be the most biocompatible [23, 40]. Bioroot RCS was compared to AH plus and ZOE in two of these studies [18, 23]. Comparing bioceramic sealers to other experimental groups, study results showed that they were superior. Studies have demonstrated apical foramen enlargement enhanced periapical healing as the disinfection of the root canal system would occur in the apical third [41, 42]. However, literature evidence in recent years has indicated that overzealous enlargement of the foramen can disrupt the apical seal. This leads to overextension of obturating material, which impedes periapical healing. Some cases where the apical foramen by itself became wider can be attributed to inadvertent extrusion of the sealer. As a result, bioceramics and bioactive sealers play a key role in minimizing acute inflammatory responses and promoting quicker periapical healing.

## 5. Conclusions

Bioactive sealers reported better periapical healing than zinc oxide eugenol, although some of the included studies were not of high-quality evidence. This aspect should be focused on in future trials to provide clear information about all the root canal sealers. Thus, compiling the results of the included studies, we infer that compared to zinc oxide eugenol, the bioactive sealers demonstrated better periapical healing. Other sealers, when compared with zinc oxide eugenol, showed similar results regarding periapical healing in a six-month follow-up.

## Figures and Tables

**Figure 1:** Search strategy framework with PRISMA 2020 guidelines.

**Figure 2:** Risk bias domain framework.

**Table 1:** Study characteristics.

*N*	Study design	Sample	Tooth type	Study groups	Clinical protocol	Outcomes	Ref
1	Random control trial (RCT)	45	Single rooted teeth	Group 1—zinc oxide eugenol (Tubliseal) Group 2—epoxy resin (AH plus) Group 3—MTA (ProRoot MTA)	Rotary (Protaper gold); 2.5% NaOCl, 17% EDTA; activation protocol not specified; two visits; calcium hydroxide medicament for 1 week; lateral compaction technique.	Postoperative pain and periapical healing	[25]
2	RCT	199	Single rooted teeth	Group 1—silicone-based sealer (Roeko Seal Automix) Group 2—zinc oxide eugenol-based sealer (Grossman's sealer)	Unclear instrumentation and irrigation protocol; two visits; calcium hydroxide medicament for 1 week; lateral compaction technique	Healing of apical periodontitis	[21]
3	RCT	204	—	Group 1—ZOE based sealer (ProcoSol) Group 2—ZOE-based sealer with incorporated calcium hydroxide (CRCS) Group 3—salicylate resin-based sealer (Sealapex)	Hand instrumentation; irrigation and activation protocol are not specified; the number of visits and type of intracanal medicament is not specified; lateral compaction technique.	Periapical healing	[22]
4	RCT	233	All teeth	Group 1—ZOE based sealer (ProcoSol) Group 2—epoxy resin-based sealer (AH26) Group 3—ResinGutta-percha-chloroform sealer (Kloroperka NO)	Hand instrumentation; 0.5% NaOCl, irrigant activation protocol was not specified; two visits; calcium hydroxide medicament at least for one week; obturation technique not specified.	Periapical healing	[19]
5	RCT	63	A single or multirooted mature tooth	Group 1: bio root RCS Group 2: pulp canal sealer (ZOE)	Rotary instrumentation up to 30 07, irrigated with 5% NaOCl. Group 1 obturated with standardized gutta-percha. Group 2 obturated with warm vertical compaction. No details were mentioned regarding the visits for root canal treatment.	Periapical healing	[24]
6	RCT	63	Maxillary anterior teeth	Group 1: ZOE based sealer Group 2: epoxy resin-based sealer (AH plus) Group 3: bioceramic-based sealer (BioRoot RCS)	Rotary instrumentation using proper gold. Preparation taper not mentioned. 3% NaOCl. Calcium hydroxide intramaedicament was placed and recalled after one week.	Periapical healing and postoperative pain	[23]
7	Clinical trial	52	Maxillary anterior teeth	Group 1: bioceramic sealer Group 2: MTA-based sealer Group 3: resin-based sealer (AH plus) Group 4: zinc oxide eugenol sealer	Type of instrumentation not mentioned. 2 ml of 2.5% NaOCl and 2.0 mL of sterile saline followed by 10 ml 17% EDTA. Obturation done in single visit.	Periapical healing and other clinical symptoms (pain, sinus tract, mobility, and swelling)	[18]
8	Clinical trial	150	—	Group 1: ProcoSol sealer Group 2: CRCS sealer Group 3: Sealapex	—	Periapical healing	[17]
9	Clinical trial	571	All teeth	Group 1: AH 26 Group 2: ProcoSol Group 3: Kloroperka	—	Periapical healing	[20]

**Table 2:** Follow up details and statistical outcomes.

*N*	Follow-up period	Loss of follow-up	Statistical analysis	Results	Sealer treatment	Ref
1	6 months	—	Wilcoxon sign rank test for intragroup comparison and intergroup comparison was done using Kruskal-Wallis test followed by Mann-Whitney *U* test.	A significant difference in PAI score was seen on comparing the baseline and 6 months. However, the difference was not evident among the groups.	All the three compared sealers showed similar healing at 6-month follow-up.	[25]
2	3-12 months	Out of 199 teeth evaluated, 43 teeth were lost for follow-up.	Mann-Whitney *U* test and Friedman's test.	The improvement in bone was 47 and around 78% at 3 and 12 months, respectively. There was a statistically significant decrease in PAI scores at both intervals. No significant difference between the groups at the start or any of the follow-ups was seen.	All the compared sealers showed similar healing at one year follow-up.	[21]
3	12 months 24-36 months 48 months	53 patients lost for follow-up 18 patients lost for follow-up 56 patients were lost for follow-up	Ridit statistic (*r*) was used to compare the PAI scores in the groups assessed.	The salicylate resin-based sealers containing calcium hydroxide showed statistically significant better periapical healing at 12 and 24 months but the results after 36 months and 48 months were statistically indistinguishable.	Calcium hydroxide containing sealers have shown better healing as compared to the other types.	[22]
4	36 months	Out of 233 teeth, 112 were lost for follow-up.	Ridit statistic (*r*) was used to compare the PAI scores in the groups assessed.	The response of Kloroperka seemed slightly inferior to others, with no statistically significant difference elicited among the assessed groups.	Healing of periapical lesions was evident after 3 years, with no difference among the compared sealer types.	[19]
5	12 months	Follow-up rate was 82%	*t*-tests for the equality of means, and nonparametric *k*-sample tests for the equality of medians was used to perform analyses	Bioceramic sealers showed better healing when compared to ZOE sealers, but were not significant	Healing of periapical lesions was evident after 12 months, with no difference.	[24]
6	6 months	6 patients reported with loss of follow-up	The Chi-square test was used to assess the difference in the extrusion rates among the groups. Mann–Whitney *U* test was used to assess the differences in the mean pain scores Kruskal-Wallis test and Friedman's two-way	Periapical healing was better in Bioroot RCS compared to AH plus and zinc oxide-based sealer at 3 and 6 months	Periapical healing was better in Bioroot RCS was better than other sealers	[23]
7	6 months	—	One-way ANOVA–F test	A significant difference was found with bioceramic sealer compared with other sealers whereas no difference found with MTA, AH plus, and ZOE	Bioceramic sealers were superior compared to other sealers	[18]
8	48 months	—	—	1^st^ year after filling, the mean credit value decreased in all test groups At 2 years, sealapex had slightly better than group CRCS and ProcoSol At 3 and 4, no difference was detectable	During the follow-up period of 4 years, no difference was found among the sealers	[17]
9	48 months	32.9% loss of follow-up till 12 months and loss of follow-up at 48 months data not reported	Chi-square analysis was performed to assess statistically significant differences among treatment groups	AH 26 and/or ProcoSol performed better than Kloroperka	During the follow-up period of 4 years, AH 26 and ProcoSol showed better healing.	[20]

## Data Availability

Data set used in the current study will be made available at the reasonable request.
